# Ferroptosis-Related Long Noncoding RNAs as Prognostic Marker for Colon Adenocarcinoma

This article has been retracted.

**DOI:** 10.1155/2022/5220368

**Published:** 2022-04-08

**Authors:** Yuting Qiu, Haobo Li, Qian Zhang, Xinwei Qiao, Jing Wu

**Affiliations:** ^1^Department of Gastroenterology, Beijing Friendship Hospital, Capital Medical University, National Clinical Research Center for Digestive Diseases, Beijing 100050, China; ^2^Graduate School of Peking Union Medical College, Chinese Academy of Medical Sciences, Beijing 100029, China

## Abstract

**Background:**

The incidence of colon adenocarcinoma (COAD) has been increasing over time. Although ferroptosis and long noncoding RNAs (lncRNAs) have been extensively reported to participate in the tumorigenesis and development of COAD, few studies have investigated the role of ferroptosis-related lncRNAs in the prognosis of COAD.

**Methods:**

Gene-sequencing and clinical data for COAD were obtained from The Cancer Genome Atlas database. The coexpression network was constructed using known ferroptosis-related genes. Cox and least absolute shrinkage and selection operator regression were used to screen ferroptosis-related lncRNAs with prognostic value and to identify a predictive model of COAD. Patients with COAD were divided into low- and high-risk groups according to their risk score. Cases of COAD in the International Cancer Genome Consortium database were included as the testing cohort.

**Results:**

In total, nine lncRNAs (LINC02381, AC105219.1, AC009283.1, LINC01011, ELFN1-AS1, EIF3J-DT, NKILA, LINC01063, and SNHG16) were considered prognostic factors for COAD. Then, a risk score model was established. The overall survival rate of COAD patients was negatively associated with the risk score. Kaplan–Meier analyses in the original and testing cohorts showed similar results. The expression of the lncRNAs in tissue was consistent with the risk score, and the relationship with tumor mutation burden, immunity, and drug sensitivity presented a marked link between the signature and COAD. A nomogram was established for clinical applications.

**Conclusions:**

Nine ferroptosis-related lncRNAs and the established signature have a certain predictive value for prognosis of COAD patients and can be used as potential research targets for exploring treatment of COAD.

## 1. Introduction

Colorectal carcinoma (CRC) is one of the most common types of cancers worldwide, with the third and second highest incidence and mortality rates, respectively [1]. Among the new cases of CRC in China in 2015, colon cancer (CC) accounted for a higher proportion than rectal and anal cancers [2]. Colon adenocarcinoma (COAD) is the most common pathological type of CC. In recent decades, the incidence of COAD has drastically increased in developing countries, such as China, with family history, old age, and unhealthy diet being considered risk factors [3, 4]. A large proportion of COAD cases follows the process from adenoma to adenocarcinoma, and patients usually have no discomfort until the disease is advanced. With the widespread use of colonoscopy, the cure rate of early-stage COAD has increased in recent decades; however, more attention has been paid to advanced COAD, especially stage III. Surgery is the preferred method for non-metastatic COAD, whereas adjuvant chemotherapy, DNA testing, and targeted therapy are recommended for advanced cases [5]. However, there is no effective way to predict the prognosis of patients with COAD. Therefore, finding a convenient and sensitive method of prediction is of great clinical value.

Ferroptosis is a newly discovered nonapoptotic form of cell death that relies on intracellular iron and is not regulated by apoptotic proteases. Morphologically, it manifests as atrophy of mitochondria, increased mitochondrial membrane density, and the decrease/disappearance of mitochondrial cristae. In biochemistry, it is characterized by the fatal accumulation of iron metabolism-related lipid reactive oxygen species (ROS), the gradual consumption of glutathione, and the inactivation of the lipid repair enzyme GPx4 [6]. Numerous studies have discovered the anticancer function of ferroptosis and its involvement in cancer therapy. Lei Shi et al. clarified that ferroptosis induced by some biological agents is involved in immunotherapy for cancer based on its function of regulating antitumor immunity, such as interfering with the immune escape of tumor cells and maintaining immune responses [7]. In particular, ferroptosis can be used for the treatment of CC. For example, Malfa et al. found that an extract of Betula aetnensis Rafin can upregulate the expression of heme oxygenase-1 (HO-1), induce ferroptosis, and result in cell death in Caco2 cell lines [8]. In addition, Li et al. applied iron-based nanomaterials to tumor therapy for a better induction effect of ferroptosis and a more efficient anticancer condition [9]. In CC, a biocompatible fusiform iron oxide-hydroxide nanospindle (FeOOH NSs) nanosystem was created by Li et al. for specific treatment, as it causes cell death via ferroptosis [10]. There is great potential for ferroptosis in tumor therapy to be explored. Therefore, clarifying the relevant mechanism of ferroptosis in CC might have important clinical significance for prognostic prediction and finding new therapeutic targets for CC.

Long noncoding RNAs (lncRNAs) are noncoding RNAs with a length > 200 nucleotides. While unable to encode proteins, lncRNAs can regulate gene expression at different levels, such as chromosome modification, transcription, and posttranscriptional translation [11]. Numerous studies have found that the abnormal regulation of lncRNAs is related to the initiation and development of a variety of diseases, especially cancer. In cancer, the competing endogenous RNA (ceRNA) model is one of its characteristic and common mechanisms; ceRNAs can promote or inhibit the development of tumors by sponging corresponding miRNAs. Many lncRNAs function as oncogenes, promote tumor growth, and are often overexpressed in cancers, whereas others might play a protective role in preventing cancer progression [12]. Furthermore, lncRNAs have been considered biomarkers for the diagnosis and prognosis of CC. Zhu et al. discovered the overexpression of BLACAT1 in CC tissues, which could facilitate the binding of EZH2 and upregulate the level of H3K27me3; BLACAT1 is an important prognostic factor of CC [13]. In addition, lncRNAs play an important role in ferroptosis. For example, lncRNA P53RRA can activate p53, a classical tumor suppressor that resides in the nucleus, triggering ferroptosis and inhibiting tumor progression [14].

Nevertheless, there is still no strong evidence for a connection among COAD, lncRNAs, and ferroptosis, and few systematic studies have focused on the relationship between ferroptosis-related lncRNAs and COAD. We hypothesized that ferroptosis is involved in the occurrence and development of COAD, and that this is linked via lncRNAs. This study is aimed at exploring the ferroptosis-related lncRNAs with prognostic value for COAD and establishes a simple and accurate signature for predicting the prognosis of COAD patients based on these lncRNAs. As COAD is one of the most common types of CRC, we believe that this model could provide a basis for further research on the specific mechanism and significance of ferroptosis in CRC and offer possible directions for determining novel therapeutic targets.

## 2. Material and Methods

### 2.1. Datasets and Sample Extraction

Gene-sequencing (gene-seq) and clinical data of COAD were obtained from The Cancer Genome Atlas (TCGA) database (https://portal.gdc.cancer.gov/repository) up to 14 February 2021 and bioinformatic analysis of 14,142 lncRNAs from 398 COAD samples were performed [15]. While screening clinical information, specific exclusion criteria for the studies were as follows: (1) patients with a survival duration of less than 30 days, as they might die of diseases other than COAD, (2) patients without integrated clinical information (age, sex, and TNM stage), and (3) lack of matching gene-seq data. Clinical data from 355 patients with COAD were evaluated. Additionally, 134 cases of COAD in the International Cancer Genome Consortium (ICGC) database (https://icgc.org/) were included as a test cohort for external validation [16]. As TCGA and ICGC data are publicly available for scientific research, no ethics approval was required. The ferroptosis-related genes were retrieved from the literature [17–20] and are presented in Supplementary Table 1.

### 2.2. Identification of a Ferroptosis-Related lncRNA Signature

First, ferroptosis-related lncRNAs were selected by Pearson correlation analysis with the coefficient of the cor − filter > 0.3 and *P* < 0.001. Univariate Cox regression was used to identify the ferroptosis-related lncRNAs with prognostic value. LncRNAs with *P* values less than 0.05 were included in least absolute shrinkage and selection operator (LASSO) regression. Next, the results of LASSO were applied to multivariate Cox regression to acquire independent prognostic ferroptosis-related lncRNAs (*P* < 0.1), which were used to construct a ferroptosis-related lncRNA signature. The risk score formula was established through a linear combination of the ferroptosis-related lncRNAs multiplied by a regression coefficient, as follows:

(1) $$\begin{array}{c} \text{Risk}\;\text{Score}=\overset{N}{\underset{i=1}{\sum }}\left(\text{Coefficient}\;\left(\text{lncRNA}i\right)\times \text{Expression}\left(\text{lncRNA}i\right)\right). \end{array}$$

Network and Sankey diagrams were used to explore the relationship between prognostic ferroptosis-related lncRNAs and mRNAs in COAD. Linear correlations were performed to validate the relationship between the prognostic ferroptosis-related lncRNAs and their corresponding mRNAs.

### 2.3. Validation of the Established Signature

The COAD patients were divided into two groups (high-risk and low-risk groups) in accordance with the median risk score. A scatter plot was constructed to determine the relationship between the survival duration and risk score. “Beeswarm” packages were used to evaluate the risk score among the deceased and living patients. The heat map demonstrates the expression of each prognostic ferroptosis-related lncRNA in each sample. We conducted a Kaplan–Meier (KM) survival curve analysis and a log-rank test to explore the difference in overall survival (OS) between the two risk groups. The same steps were then applied to the testing cohort for external validation. Receiver operating characteristic (ROC) curves and the area under the curve (AUC) were applied to explore the sensitivity and specificity of the signature in both cohorts [21]. Furthermore, KM curve analyses of each prognostic ferroptosis-related lncRNA were carried out to explore the difference in OS between the high- and low-expression groups.

### 2.4. Prognostic Value of the Ferroptosis-Related lncRNA Signature

We performed univariate and multivariate Cox regression analyses to clarify whether the risk score was an independent predictive factor of OS in COAD patients by adjusting for the influence of age, sex, TNM pathological stage, and body mass index (BMI).

### 2.5. Clinical Application of the Ferroptosis-Related lncRNA Signature

A nomogram was generated for survival rate prediction for COAD patients. The index of concordance (*C*-index), ROC curves, and calibration curves was applied to evaluate the congruency between predicted and actual survival.

### 2.6. Test of Expression of Ferroptosis-Related lncRNAs in Tissues

The ICGC database was used to analyze the differences in the lncRNA expression between COAD and normal tissues.

### 2.7. Functional Analysis

To explore the potential functions of the constructed signature, Kyoto Encyclopaedia of Genes and Genomes (KEGG) analysis was conducted using gene set enrichment analysis (GSEA 4.1.0). Functional enrichment of ferroptosis-related lncRNAs was investigated, and the top five KEGG signal pathways were visualized in high- and low-risk groups.

### 2.8. Relationship with Tumor Mutation Burdens (TMB), Immune, and Drug Sensitivity

A mutation profile of the top 15 genes with the highest mutation frequency was drawn using the “maftools” package. We compared seven algorithms to show immune responses in samples between high- and low-risk groups based on ferroptosis-related signatures. Single-sample GSEA was then used to determine the infiltrating score of immune cells, functions, and checkpoint gene expression between the two groups. The half-maximal inhibitory concentration (IC50) of chemotherapy drugs in each COAD sample from TCGA database was estimated with the Genomics of Drug Sensitivity in Cancer (GDSC) database using the “pRRophetic” package. The differences in TMB and drug sensitivity for samples between the high- and low-risk groups were analyzed using the Wilcoxon test.

### 2.9. Statistical Analysis

We utilized *R* version 3.6.0 software (https://www.r-project.org/) and Perl version 5.32.0.1 software (https://www.perl.org/) for statistical analyses. Heat maps were generated with the “pheatmap” package, and KM survival analyses were performed with “survival,” “survminer,” and “timeROC” to generate the survival curves. Statistical tests were bilateral, and statistical significance was set at *P* < 0.05.

## 3. Results

Ferroptosis has been shown to play a significant role in various cancers. Additionally, lncRNAs are considered indispensable in both cancers and ferroptosis. We hypothesized that ferroptosis is involved in the occurrence and development of COAD, linked via lncRNAs. This study was thus conducted to clarify the relationship among ferroptosis, COAD, and lncRNAs. We constructed a coexpression network of ferroptosis-related genes and lncRNAs and placed these lncRNAs successively into univariate Cox, LASSO, and multivariate Cox regression analyses. Finally, the ferroptosis-related lncRNAs with independent prognostic value for COAD were selected, and their signature was identified. The prognostic value of the signature was validated in both internal and external cohorts and in clinical tissues. A nomogram was developed for clinical application, and function analysis was also conducted. The workflow of the research is shown in Figure S1.

### 3.1. Data Collection and Construction of Coexpression Network

First, gene-seq data, including 14,142 lncRNAs of 398 COAD samples, were obtained from TCGA-COAD. We then collected clinical information of 385 COAD patients in the same database, 26 of which were excluded for a follow-up time of less than 30 days and four for the absence of RNA-seq. Clinical data from 355 COAD patients were collected. Second, 60 genes related to ferroptosis were identified from previous literature (Table S1) [17–20], of which 59 were expressed in COAD (Table S2). Third, a Pearson correlation analysis was performed between the 59 ferroptosis-related genes and lncRNAs of COAD from TCGA. The lncRNAs with a coefficient of the cor − filter > 0.3 and *P* < 0.001 were selected as ferroptosis-related lncRNAs, and the coexpression network combining ferroptosis-related genes and lncRNAs expressed in COAD was constructed.

### 3.2. Filtration of Prognostic Ferroptosis-Related lncRNAs and Identification of a Ferroptosis-Related lncRNA Signature

To identify the prognostic value of the ferroptosis-related lncRNAs, univariate Cox regression analysis was utilized, leading to the identification of 29 ferroptosis-related lncRNAs (Table S3, *P* < 0.05). LASSO regression further identified 15 ferroptosis-related lncRNAs from the above list (Figure S2). Finally, multivariate Cox regression analysis identified nine lncRNAs that have independent prognostic value (*P* < 0.1, Figure S3, Table 1). Among them, eight lncRNAs (LINC02381, AC105219.1, AC009283.1, LINC01011, ELFN1-AS1, EIF3J-DT, NKILA, and LINC01063) were considered harmful prognostic factors, given that the hazard ratio (HR) of these lncRNAs was >1, and one lncRNA (SNHG16) was considered a protective factor with an HR < 1. The ferroptosis-related lncRNA signature was established, and the formula was defined as risk score = (0.42031 × LINC02381) + (0.12636 × AC105219.1) + (0.05421 × AC009283.1) + (0.52185 × LINC01011) + (0.02171 × ELFN1 − AS1) + (0.32914 × EIF3J − DT) + (0.18289 × NKILA) + (0.53534 × LINC01063) − (0.14385 × SNHG16). At the same time, network and Sankey diagrams were provided for the visualization of these lncRNAs and related mRNAs (Figures 1(a) and 1(b), Figure S4).

### 3.3. Validation of the Established Signature

In light of the risk score, we divided the patients into high- and low-risk groups (Figure 2(a)). As portrayed in Figure 2(b), the survival time decreased as the risk score increased. Moreover, the distribution of the risk score was confirmed to be statistically significant among the deceased and living groups (Figure 2(c)). The heat map of the expression of nine ferroptosis-related lncRNAs intuitively demonstrated that harmful factors were expressed at a higher level in the high-risk group, whereas a protective factor was higher in the low-risk group (Figure 2(d)). The survival time of patients in the low-risk group was longer than that in the high-risk group, which was in accordance with the KM survival curve of risk score, suggesting that the risk score based on the nine lncRNAs was negatively associated with the OS of the COAD patients (Figure 3(a)*P* < 0.05). We also conducted the same steps for external validation. The results revealed that the signature still had considerable predictive value, with a *P* value <0.05, in the testing groups (Figure 3(c)*P* < 0.05, Table S4). The AUCs for survival times of 1, 3, and 5 years in the original and testing cohorts were 0.701, 0.785, 0.821, 0.701, 0.751, and 0.833, respectively, which indicated both the accuracy of the signature and that it had a relatively higher value for 5-year survival (Figures 3(b) and 3(d)). The KM survival curve of each lncRNA is provided in Figure S5. The results were consistent with the aforementioned conclusion, and the *P* value for each lncRNA was less than 0.05, suggesting that the expression of each lncRNA had a significant impact on the OS of COAD patients.

### 3.4. Prognostic Value of the Ferroptosis-Related lncRNA Signature

Univariate and multivariate Cox regression analyses were used to examine the prognostic value of the ferroptosis-related lncRNA signature. Univariate analysis revealed that the risk score and stage were independent prognostic factors for COAD (Table S5, *P* < 0.001). The HR of the risk score was 3.268 (95% CI: 1.948–5.482, Figure 4(a)). Multivariate Cox regression was applied, and the risk score turned out to be an independent prognostic biomarker (*P* < 0.001, HR = 2.457, 95% CI: 1.418–4.257, Figure 4(b), Table 2), which was similar when adjusted based on the clinical features. BMI showed a correlation with prognosis; however, it was not strong. This indicates that obesity might not be a risk factor for poor outcome of COAD. In summary, the outcomes indicated the excellent predictive value of the ferroptosis-related lncRNA signature for predicting the prognosis of patients with COAD.

### 3.5. Clinical Applications of the Ferroptosis-Related lncRNA Signature

A nomogram including age, stage, and risk score was designed for clinical application (Figure 5(a)). The risk score showed a strong predictive value for survival. The *C*-index was 0.801 (95% CI: 0.769–0.833), and the AUC of the 5-year survival rate was 0.821 for the model, which confirmed the predictive ability of the signature (Figure 5(b)). The nomogram-predicted probability of 5-year OS also showed considerable consistency with the actual 5-year OS (Figure 5(c)). The risk score increased with increasing stage (Table 3). Taken together, these data suggest that the nine ferroptosis-related lncRNAs might be related to the development of COAD.

### 3.6. Expression of Ferroptosis-Related lncRNAs in COAD and Normal Tissues

We then tested the expression of each ferroptosis-related lncRNA with the information of COAD tumor tissue and normal tissue supplied in the ICGC database. As expected, all of the harmful prognostic lncRNAs (LINC02381, AC105219.1, AC009283.1, LINC01011, ELFN1-AS1, EIF3J-DT, NKILA, and LINC01063) were expressed at higher levels in tumor tissues than in normal tissues (Figure 6). The results confirmed the prognostic value of the model at the clinical level.

### 3.7. Function Analysis

GSEA was performed to identify potential signaling pathways that involved the nine ferroptosis-related lncRNAs. In total, 178 KEGG pathways were acquired in both the high- and low-risk groups, and these lncRNAs were mainly enriched in tumor-related pathways. The enriched signaling pathways were ranked according to the nominal *P* value in each group (Figure 7(a), Table S6). In the high-risk group, “GLYCOSAMINOGLYCAN_BIOSYNTHESIS_CHONDROITIN_SULFATE” was the top-ranked pathway, followed by “SNARE_INTERACTIONS_IN_VESICULAR_TRANSPORT,” “HEDGEHOG_SIGNALING_PATHWAY,”,“ECM_RECEPTOR_INTERACTION,” and “BASAL_CELL_CARCINOMA” (Figure 7(b)). In the low-risk group, the lncRNAs were mainly enriched in energy metabolism, including “CITRATE_CYCLE_TCA_CYCLE,” “FRUCTOSE_AND_MANNOSE_METABOLISM,” “GLYCOLYSIS_GLUCONEOGENESIS,” “PORPHYRIN_AND_CHLOROPHYLL_METABOLISM,” and “FATTY_ACID_METABOLISM” (Figure 7(c)). Most of the signaling pathways listed have been reported to contribute to tumor progression. These results further validate the predictive value of the lncRNA signature and suggest the potential molecular mechanisms of COAD.

### 3.8. Relationship with TMB, Immune, and Drug Sensitivity

Fifteen genes in each of the high- and low-risk groups that showed the highest mutation frequency were selected (Figure 8(a)). The majority of these genes were shared between both groups, including several classical genes known to be involved in CC (APC, TP53, and KRAS). The mutation frequency of the top two genes, APC and TP53, was higher in the high-risk group. Additionally, TMB in the high-risk group was also significantly higher (Figure 8(b)). We designed a heat map to show the immunity responses obtained based on the seven algorithms and evaluated their correlation with immune cells and functions in high- and low-risk groups (Figures 8(c)–8(e)). The expression of genes associated with dendritic cells and Th1 and Th2 cells was significantly higher in the low-risk group. Similarly, immune functions, including chemokine receptor (CCR), antigen-presenting cells (APC) costimulation, and cytolytic activity, were also higher in the low-risk group. Furthermore, the immune checkpoints TNFSF9 and ICOS were found to be higher in the low-risk group (Figure 8(f)). The results of drug sensitivity prediction illustrated that there was a significant difference in the estimated IC50 between the two groups, and the patients in the low-risk groups had a more sensitive response to common chemotherapy (Figures 8(g)–8(i)).

## 4. Discussion

COAD is the most common type of CC, which accounts for a large proportion of CRC. There have been an increasing number of treatments for COAD, especially for stage III patients and not only treatments recommended by guidelines like adjuvant chemotherapy and targeted therapy but also some traditional agents with newly discovered anti-cancer effects, such as polysaccharides and prostaglandin E2 [22–24]. Carcinoembryonic antigen is a confirmed marker for predicting the prognosis of COAD, whereas its accuracy is limited. Some new biomarkers of COAD have also been reported, such as proteins like cytoplasmic aspirin or miRNAs like extracellular vesicle-derived miR-139-3p and miR-145-3p, among others [25, 26]. However, there is still lack of evidence regarding their predictive value for COAD.

Ferroptosis can disturb various mechanisms of tumor development, such as immune evasion and tumor angiogenesis, and nanoformulations might be a novel direction for tumor treatment [7, 27]. It has been gradually acknowledged that lncRNAs are significant regulators of ferroptosis. Based on the hypothesis that ferroptosis-related lncRNAs would have prognostic value for predicting the progression of COAD, we obtained RNA-seq data of COAD from TCGA and ferroptosis-related genes from previous literature [17–20] and performed regression analyses on these datasets, leading to the identification of a total of nine ferroptosis-related lncRNAs that might have prognostic value for COAD.

Five ferroptosis-related lncRNAs (ELFN1-AS1, EIF3J-DT, LINC01063, LINC02381, and LINC01011) were thought to be CC-related, and their influence on tumor progression, as shown by previous studies, was consistent with our results. Most of them were proven to function as ceRNAs, similar to how lncRNAs accelerate tumor progression. ELFN1-AS1 has been observed to be overexpressed in various types of cancers, including CC, and has a negative effect on good prognosis. It was selected as a lncRNA with prognostic value in CC in previous bioinformatic analyses, and its functions in tumor proliferation and invasion were further explored by Du et al. [28, 29]. Liu et al. found that the EIF3J-DT expression is upregulated in CRC tissues and cell lines and has a negative relationship with good prognosis, suggesting that EIF3J-DT is a carcinogenic factor in CRC. It inhibits tumor cell apoptosis and is a therapeutic target for CRC [30]. LINC01063 also possesses carcinogenetic functions and is part of the autophagy-related lncRNA signature in COAD. The overexpression of LINC01063 might correspond with tumor metastasis [31]. LINC02381 is an oncogenic factor in several lncRNA signatures and indicates a poor prognosis for CC [31, 32]. LINC01011 is also considered a stimulator of COAD as reported in another study revealing an autophagy-related lncRNA signature [31].

Interestingly, there were two ferroptosis-related lncRNAs (NKILA and SNHG16) that had opposite effects on cancers in previous studies. A meta-analysis and functional experiments on NKILA found low expression of NKILA in CC and resulted in a poor prognosis, which suggested that NKILA has a protective function in CC cell lines and tissues. This is opposite to our results [33, 34]. However, Huang et al. found that NKILA could strengthen the sensitivity of tumor-specific cytotoxic T lymphocytes and TH1s to activation-induced cell death and help in the immune escape of tumor cells, suggesting that it is a risk factor, which is consistent with our results [35]. In contrast to our results, SNHG16, which has been widely studied, was found to be a carcinogenetic factor for CC. It promotes cell proliferation and tumor development and was linked to poor prognosis [36, 37]. Additionally, the expression of SNHG16 was higher in tumor tissues in ICGC database in this study. However, SNHG16 mainly influences genes related to lipid metabolism and can inhibit oxidative stress-induced pathological angiogenesis. We hypothesized that SNHG16 might have a similar protective effect in COAD cells, which is different from what is known about this gene [38, 39]. This might reveal some new links between ferroptosis and COAD and could be a target for further study.

As for the other two lncRNAs (AC009283.1 and AC105219.1), no studies on their prognostic value in CRC have been performed. Therefore, it is essential to investigate the mechanism by which lncRNAs influence COAD prognosis through ferroptosis. Moreover, some of the lncRNAs seemed to have dual effects on different cancers; therefore, their exact mechanisms should be explored with more functional experiments.

A risk score model of nine ferroptosis-related lncRNAs was constructed to predict the survival of COAD patients, and the time-dependent ROC analysis presented had predictive value, especially for long-term survival (5-year OS). Many other risk score models of lncRNAs have been identified for CRC and CC [40–42]. We compared the AUC for the 5-year OS of this signature (0.821) with those of previous studies (0.674, 0.731, and 0.739, respectively), and the ferroptosis-related signature was significantly superior to the others. Additionally, this study focused on a subtype of CC (COAD) and a specific mechanism (ferroptosis), which might also improve the accuracy of the signature to some extent and lead to future studies on ferroptosis in COAD. A nomogram was designed for clinical applications. The results of statistical analyses revealed that the signature exhibited good discriminative potential and accuracy. We also checked the expression of each ferroptosis-related lncRNA in tumor and normal tissues, and the results further confirmed the value of this model. While considering the prognostic value of the risk score combined with other clinical characteristics, obesity turned out not to be a risk factor for COAD. However, Friedenreich et al. has stated that obesity is associated with an increased risk of CRC [43]. Therefore, it is necessary to further explore the relationship between COAD prognosis and obesity.

GSEA was conducted to detect the probable molecular mechanisms underlying the functions these lncRNAs, and several KEGG signaling pathways were selected. In the high-risk group, the lncRNAs were mostly enriched in the glycosaminoglycan (GAG) biosynthesis-chondroitin sulphate (CS) pathway. CS is a GAG that has anti-inflammatory properties. Lipid peroxidation, which is widely accepted to be a characteristic of ferroptosis, was significantly inhibited after treatment with CS in a previous study. The results revealed that CS inactivates antioxidant enzymes and inhibits ferroptosis [44]. In CC, CS content was found to be substantially increased, and the proportion of chondroitin-6-sulphate (C-6-S), which has a stronger anti-inflammatory function, was particularly elevated. This acts as a regulator of cytokines/chemokines, accelerates the production of ROS, and results in poor prognosis [45]. In summary, CS inhibits ferroptosis and promotes cancer progression. The role of glycosylation in CC was also confirmed in other researches [46]. The remaining pathways in which the lncRNAs were enriched, such as the ECM-receptor interaction, the Hedgehog (Hh) signaling pathway, and pathways involved in the development of basal cell carcinoma showed a strong relationship with cancer progression and ferroptosis. The ECM-receptor interaction pathway has been confirmed to play an important role in diverse steps of tumor progression. For example, as an extracellular matrix protein, matrix Gla protein can promote an increase in the intracellular free Ca2+ concentration and activate the NF-*κ*B pathway, which comprise a part of the mechanism underlying ferroptosis, and finally result in CC proliferation [46]. The Hh signaling pathway is also a typical pathway in tumor progression. Hh signaling regulates the morphogenesis of a variety of organs and is also involved in the control of stem cell proliferation in adult tissues [47]. The development of basal cell carcinoma is associated with constitutive activation of the sonic hedgehog signaling pathway. In the low-risk group, the lncRNAs were mainly enriched in metabolism-related pathways, including fatty acid metabolism, which might also provide some evidence of the inhibitory effect of ferroptosis on COAD.

Analyses of the differences in TMB, immunity, and sensitivity to antitumor drugs between high- and low-risk groups were in favor of the prognostic predictive value of the signature. The top two genes with the highest mutation frequency were typical mutated genes in CC, according to previous studies [4]. The checkpoints TNFSF9 and ICOS, which were expressed at significantly higher levels in the low-risk group, might become potential targets for immunotherapy. In addition, patients at a low risk showed greater sensitivity to some antitumor drugs (axitinib, metformin, and sorafenib), which have been proven to be effective in CC treatment.

Bioinformatic analyses have been widely utilized to construct models for different purposes [48]. There have been many models of lncRNAs regarding the prognosis of CC. For example, Wang et al. developed a 15-gene signature for predicting the prognosis of advanced CRC. Signatures of immune or autophagy-related lncRNAs were also generated [32, 49]. As a novel type of cell death, ferroptosis has been found to be involved in an increasing number of diseases, including COAD, and has shown great potential for tumor therapy. Therefore, it is necessary to elucidate the molecular mechanisms and pathways associated with ferroptosis in COAD. In this study, we identified nine ferroptosis-related lncRNAs in COAD and constructed a signature for prognostic prediction. We also detected several signaling pathways that are likely related to ferroptosis in COAD. This might provide possible directions for future research and help to determine potential treatment targets for COAD. A few limitations still existed in our research as follows: (1) the statistics applied were all from public databases, and they might not reflect authentic clinical conditions. Additionally, data in public databases are limited to the comprehensive study of the disease. Our study could thus represent a preliminary study, and further prospective studies are required to confirm the value of the selected lncRNAs. (2) Further, the numbers of ferroptosis-related genes revealed by RNA-seq were not large enough to control for deviation in an ideal range. (3) Moreover, since the signature of lncRNAs was validated using only two datasets, the robustness might not be satisfactory, and we could not confirm its prognostic accuracy in wider ranges. (4) Finally, with only bioinformatic analyses, the true underlying mechanisms cannot be revealed, and these should be supplemented with further functional experiments to confirm the links between these lncRNAs and COAD.

## 5. Conclusion

In this study, nine ferroptosis-related lncRNAs and the established signature had a certain predictive value for the prognosis of COAD patients, and the nomogram designed could be applied in clinical settings. Furthermore, lncRNAs might be valuable for the future exploration of ferroptosis in COAD, and the results could be used as potential research targets for the development and treatment of COAD.

## Figures and Tables

**Figure 1:** The network and Sankey diagram of ferroptosis-related lncRNAs with prognostic value. (a) The network between prognostic lncRNAs and ferroptosis-related genes in COAD. Red ellipses represent lncRNAs, and sky-blue rectangles represent ferroptosis-related genes. (b) Sankey diagram which showed the link between prognostic lncRNAs, ferroptosis-related genes, and their risk types.

**Figure 2:** Survival analysis of COAD patients between high- and low-risk groups. (a) The high-risk group and the low-risk group divided by risk score. (b) The survival time of the COAD patients. (c) Distribution of the risk score among dead and alive patients. (d) Heat map of nine ferroptosis-related lncRNAs level in each patient. The color from green to red represents a rising tendency from low to high expression.

**Figure 3:** Validation of the risk score model in original and testing COAD cohorts. (a) The KM survival curve of COAD patients in two groups in original cohort. (b) The time-dependent ROC curve and the AUC about 1 year, 3 years, and 5 years in original cohort. (c) The KM survival curve of COAD patients in two groups in testing cohort. (d) The time-dependent ROC curve and the AUC about 1 year, 3 years, and 5 years in testing cohort.

**Figure 4:** Independent prognostic predictive value of the nine ferroptosis-related lncRNAs based signature. (a) The forest plots for univariate Cox regression analysis in COAD patients. (b) The forest plots for multivariate Cox regression analysis in COAD patients.

**Figure 5:** The clinical application of the nine ferroptosis-related lncRNA-based signature. (a) A nomogram to predict the survival rate of patients with COAD. (b) The ROC curves analysis based on risk score and other parameters. (c) Calibration plots for assessing the consistence between the predicted and the actual survival rate for the signature.

**Figure 6:** Expression levels of ferroptosis-related lncRNAs in COAD samples and normal samples from ICGC database. (a) ELFN1-AS1. (b) EIF3J-DT. (c) LINC01063. (d) LINC02381. (e) LINC01011. (f) AC009283.1. (g) NKILA. (h) AC105219.1.

**Figure 7:** Functional enrichment of the nine ferroptosis-related lncRNAs. (a) The KEGG enrichment scores in the high-risk group and low-risk group. (b) KEGG enriched pathways in the high-risk group. (c) KEGG enriched pathways in the low-risk group.

**Figure 8:** (a) Distribution of frequently mutated genes in high- and low-risk groups. (b) Comparison of TMB between high- and low-risk groups in the TCGA-COAD cohort. (c) The heat map of immune responses between high- and low-risk groups. (d) ssGSEA scores of immune cells. (f) ssGSEA scores of immune functions. (g) Differences in the expression levels of immune checkpoints. (h) Estimated IC50 values of axitinib, metformin, and sorafenib for tumor cells from high- and low-risk groups. Adjusted *P* values were showed as ^∗^*P* < 0.05; ^∗∗^*P* < 0.01; ^∗∗∗^*P* < 0.001.

**Table 1:** Multivariate Cox results of lncRNAs based on TCGA-COAD data.

lncRNA	Coefficient	HR	95% CI of HR	*P* value
AC009283.1	0.054	1.056	1.012-1.101	0.011
AC105219.1	0.126	1.135	0.977-1.318	0.097
EIF3J-DT	0.329	1.390	1.048-1.843	0.022
ELFN1-AS1	0.022	1.022	0.997-1.048	0.091
LINC01011	0.522	1.685	1.137-2.497	0.009
LINC01063	0.535	1.708	1.199-2.432	0.003
LINC02381	0.420	1.522	1.252-1.851	<0.001
NKILA	0.183	1.201	1.039-1.388	0.013
SNHG16	-0.144	0.866	0.740-1.014	0.073

Abbreviations: HR: hazard ratio; CI: confidence interval.

**Table 2:** Multivariate Cox regression results of risk score and clinical characteristics of COAD patients.

Variable	*B*	SE	*Z*	HR	95% CI of HR	*P* value
Age	0.036	0.012	3.031	1.037	1.013-1.062	0.002
Gender	-0.030	0.273	-0.109	0.971	0.569-1.656	0.913
Stage	0.708	0.416	1.704	2.031	0.899-4.586	0.088
T	0.118	0.308	0.385	1.126	0.616-2.058	0.701
M	0.398	0.565	0.704	1.489	0.492-4.507	0.481
N	0.045	0.263	0.171	1.046	0.624-1.752	0.864
Risk score	0.899	0.280	3.205	2.457	1.418-4.257	0.001

Abbreviations: SE: standard error; HR: hazard ratio; CI: confidence interval.

**Table 3:** Clinical influences of risk score signature for TCGA-COAD data.

Clinical	*N*	Risk score		*t*	*P*
		Mean	SD		
Age					
<70	196	2.233	6.128	2.050	0.042
≥70	159	1.292	1.757		
Gender					
Female	162	1.406	1.722	-1.600	0.111
Male	193	2.152	6.192		
Stage					
I-II	204	1.146	1.406	-2.719	0.007
III-IV	151	2.710	6.964		
T					
T1-2	74	0.996	0.732	-3.162	0.002
T3-4	281	2.026	5.273		
M					
M0	304	1.470	3.202	-1.767	0.083
M1	51	3.848	9.523		
N					
N0	211	1.128	1.387	-2.805	0.006
N1-2	144	2.813	7.116		

Abbreviations: SD: standard deviation.

## Data Availability

The data that support the findings of this study are openly available in the TCGA at https://portal.gdc.cancer.gov/repository and ICGC at https://icgc.org/.

## Supplementary Materials

Supplementary Materials Figure S1: the workflow of the research. Figure S2: ferroptosis-related lncRNA selection utilizing the LASSO model. (a) LASSO coefficient values of 15 ferroptosis-related lncRNAs in COAD. (B) Profiles of LASSO coefficients. Figure S3: multivariate Cox results of lncRNAs based on TCGA-COAD data. Figure S4: the correlation analysis of the ferroptosis-related lncRNAs and their corresponding mRNAs. Figure S5: the KM survival curves of each prognostic ferroptosis-related lncRNA. Table S1: ferroptosis-related genes retrieved from the literature. Table S2: ferroptosis-related genes expressed in COAD. Table S3: univariate cox results of ferroptosis-related lncRNAs based on TCGA-COAD data. Table S4: patients from ICGC database for external validation. Table S5: univariate Cox regression results of risk score and clinical characteristics of COAD. Table S6: gene set enrichment KEGG analysis results according to the signature of nine ferroptosis-related lncRNAs.

## References

[1] Bray F., Ferlay J., Soerjomataram I., Siegel R. L., Torre L. A., Jemal A. (2018). Global cancer statistics 2018: GLOBOCAN estimates of incidence and mortality worldwide for 36 cancers in 185 countries. *CA: a Cancer Journal for Clinicians*.

[2] Wang H., Cao M. D., Liu C. C. (2020). Disease burden of colorectal cancer in China: any changes in recent years?. *Zhonghua liu Xing Bing xue za zhi= Zhonghua Liuxingbingxue Zazhi*.

[3] Feng R. M., Zong Y. N., Cao S. M., Xu R. H. (2019). Current cancer situation in China: good or bad news from the 2018 global cancer statistics?. *Cancer Communications*.

[4] Cappell M. S. (2008). Pathophysiology, clinical presentation, and management of colon cancer. *Gastroenterology Clinics of North America*.

[5] Benson A. B., Venook A. P., Al-Hawary M. M. (2018). NCCN guidelines insights: colon cancer, version 2.2018. *Journal of the National Comprehensive Cancer Network*.

[6] Xie Y., Hou W., Song X. (2016). Ferroptosis: process and function. *Cell Death and Differentiation*.

[7] Shi L., Liu Y., Li M., Luo Z. (2021). Emerging roles of Ferroptosis in the tumor immune landscape: from danger signals to anti-tumor immunity. *The FEBS Journal*.

[8] Malfa G. A., Tomasello B., Acquaviva R. (2019). Betula etnensis Raf. (Betulaceae) extract induced HO-1 expression and ferroptosis Cell Death in Human Colon Cancer Cells. *International Journal of Molecular Sciences*.

[9] Li Y., Wei X., Tao F. (2021). The potential application of nanomaterials for ferroptosis-based cancer therapy. *Biomedical Materials*.

[10] Li Y., Chen W., Qi Y. (2020). H2S‐Scavenged and Activated Iron Oxide‐Hydroxide Nanospindles for MRI‐Guided Photothermal Therapy and Ferroptosis in Colon Cancer. *Small*.

[11] Xing J., Liu H., Jiang W., Wang L. (2021). LncRNA-encoded peptide: functions and predicting methods. *Frontiers in Oncology*.

[12] Slack F. J., Chinnaiyan A. M. (2019). The role of non-coding RNAs in oncology. *Cell*.

[13] Zhu M., Li X., Zhu S., Li P., Min L., Zhang S. (2020). Long non-coding RNA BLACAT1, a novel promising biomarker and regulator of human cancers. *Biomedicine & Pharmacotherapy*.

[14] Mao C., Wang X., Liu Y. (2018). A G3BP1-interacting lncRNA promotes ferroptosis and apoptosis in cancer via nuclear sequestration of p53. *Cancer Research*.

[15] Tomczak K., Czerwińska P., Wiznerowicz M. (2015). The cancer genome atlas (TCGA): an immeasurable source of knowledge. *Contemporary Oncology*.

[16] Zhang J., Bajari R., Andric D. (2019). The international cancer genome consortium data portal. *Nature Biotechnology*.

[17] Stockwell B. R., Friedmann Angeli J. P., Bayir H. (2017). Ferroptosis: a regulated cell death nexus linking metabolism, redox biology, and disease. *Cell*.

[18] Hassannia B., Vandenabeele P., Vanden B. T. (2019). Targeting Ferroptosis to iron out cancer. *Cancer Cell*.

[19] Bersuker K., Hendricks J. M., Li Z. (2019). The CoQ oxidoreductase FSP1 acts parallel to GPX4 to inhibit ferroptosis. *Nature*.

[20] Doll S., Freitas F. P., Shah R. (2019). FSP1 is a glutathione-independent ferroptosis suppressor. *Nature*.

[21] Blanche P., Dartigues J. F., Jacqmin-Gadda H. (2013). Estimating and comparing time-dependent areas under receiver operating characteristic curves for censored event times with competing risks. *Statistics in Medicine*.

[22] Labianca R., Beretta G. D., Kildani B. (2010). Colon cancer. *Critical Reviews in Oncology/Hematology*.

[23] Ji X., Peng Q., Wang M. (2018). Anti-colon-cancer effects of polysaccharides: a mini-review of the mechanisms. *International Journal of Biological Macromolecules*.

[24] Karpisheh V., Nikkhoo A., Hojjat-Farsangi M. (2019). Prostaglandin E2 as a potent therapeutic target for treatment of colon cancer. *Prostaglandins & Other Lipid Mediators*.

[25] Li H., Zhang Z., Chen L. (2019). Cytoplasmic asporin promotes cell migration by regulating TGF-*β*/Smad2/3 pathway and indicates a poor prognosis in colorectal cancer. *Cell Death & Disease*.

[26] Min L., Zhu S., Chen L. (2019). Evaluation of circulating small extracellular vesicles derived miRNAs as biomarkers of early colon cancer: a comparison with plasma total miRNAs. *Journal of Extracellular Vesicles*.

[27] Lopes-Coelho F., Martins F., Hipólito A. (2021). The activation of endothelial cells relies on a ferroptosis-like mechanism: novel perspectives in management of angiogenesis and cancer therapy. *Frontiers in Oncology*.

[28] Chen M., Fan M., Yang J., Lang J. (2020). Identification of potential oncogenic long non-coding RNA set as a biomarker associated with colon cancer prognosis. *Journal of Environmental Pathology, Toxicology and Oncology*.

[29] Du Y., Hou Y., Shi Y., Liu J., Li T. (2021). Long non-coding RNA ELFN1-AS1 promoted colon cancer cell growth and migration via the miR-191-5p/special AT-rich sequence-binding protein 1 Axis. *Frontiers in Oncology*.

[30] Liu D., Zhang H., Cong J. (2020). H3K27 acetylation-induced lncRNA EIF3J-AS1 improved proliferation and impeded apoptosis of colorectal cancer through miR-3163/YAP1 axis. *Journal of Cellular Biochemistry*.

[31] Zhou W., Zhang S., Li H. B. (2020). Development of prognostic indicator based on autophagy-related lncRNA analysis in colon adenocarcinoma. *BioMed Research International*.

[32] Li Z., Wang D., Yin H. (2020). A seven immune-related lncRNA signature predicts the survival of patients with colon adenocarcinoma. *American Journal of Translational Research*.

[33] Tian S., Yu Y., Huang H., Xu A., Xu H., Zhou Y. (2020). Expression level and clinical significance of NKILA in human cancers: a systematic review and meta-analysis. *BioMed Research International*.

[34] Jafari D., Noorbakhsh F., Delavari A. (2020). Expression level of long noncoding RNA NKILA-miR103-miR107 inflammatory axis and its clinical significance as potential biomarker in patients with colorectal cancer. *Journal of Research in Medical Sciences : The Official Journal of Isfahan University of Medical Sciences*.

[35] Huang D., Chen J., Yang L. (2018). NKILA lncRNA promotes tumor immune evasion by sensitizing T cells to activation-induced cell death. *Nature Immunology*.

[36] Yang M., Wei W. (2019). SNHG16: A novel long-non coding RNA in human cancers. *Oncotargets and Therapy*.

[37] Ke D., Wang Q., Ke S., Zou L., Wang Q. (2020). Long-non coding RNA SNHG16 supports colon cancer cell growth by modulating miR-302a-3p/AKT axis. *Pathology Oncology Research*.

[38] Christensen L. L., True K., Hamilton M. P. (2016). SNHG16 is regulated by the Wnt pathway in colorectal cancer and affects genes involved in lipid metabolism. *Molecular Oncology*.

[39] Zhang R., Ma X., Jiang L. (2021). Decreased lncRNA SNHG16 accelerates oxidative stress induced pathological angiogenesis in human retinal microvascular endothelial cells by regulating miR-195/mfn 2 axis. *Current Pharmaceutical Design*.

[40] Liu Y., Liu B., Jin G. (2019). An integrated three-long non-coding RNA signature predicts prognosis in colorectal cancer patients. *Frontiers in Oncology*.

[41] Fan Q., Liu B. (2018). Discovery of a novel six-long non-coding RNA signature predicting survival of colorectal cancer patients. *Journal of Cellular Biochemistry*.

[42] Li W., Yu W., Jiang X. (2020). The construction and comprehensive prognostic analysis of the LncRNA-Associated competitive endogenous RNAs network in colorectal cancer. *Frontiers in Genetics*.

[43] Friedenreich C. M., Ryder-Burbidge C., McNeil J. (2021). Physical activity, obesity and sedentary behavior in cancer etiology: epidemiologic evidence and biologic mechanisms. *Molecular Oncology*.

[44] Seol B. G., Kim J. H., Woo M. (2020). Skate cartilage extracts containing chondroitin sulfate ameliorates hyperlipidemia-induced inflammation and oxidative stress in high cholesterol diet-fed LDL receptor knockout mice in comparison with shark chondroitin sulfate. *Nutrition Research and Practice*.

[45] Pudełko A., Wisowski G., Olczyk K., Koźma E. M. (2019). The dual role of the glycosaminoglycan chondroitin-6-sulfate in the development, progression and metastasis of cancer. *The FEBS Journal*.

[46] Gao G., Li C., Fan W. (2021). Brilliant glycans and glycosylation: Seq and ye shall find. *International Journal of Biological Macromolecules*.

[47] Li X., Wei R., Wang M. (2020). MGP promotes colon cancer proliferation by activating the NF-*κ*B pathway through upregulation of the calcium signaling pathway. *Molecular Therapy-Oncolytics*.

[48] Katoh Y., Katoh M. (2005). Hedgehog signaling pathway and gastric cancer. *Cancer Biology & Therapy*.

[49] Qiu Y., Li H., Xie J., Qiao X., Wu J. (2021). Identification of ABCC5 among ATP-binding cassette transporter family as a new biomarker for hepatocellular carcinoma based on bioinformatics analysis. *International Journal of General Medicine*.

